This article has been retracted.

# Preliminary Study on Grading Diagnosis of Early Knee Osteoarthritis by Shear Wave Elastography

**DOI:** 10.1155/2022/4229181

**Published:** 2022-08-09

**Authors:** Xiaojing Zhang, Danchun Lin, Jiatong Jiang, Zexing Guo

**Affiliations:** ^1^Department of Ultrasound Medicine at the Affiliated People's, Hospital of Fujian, University of Traditional Chinese Medicine, Fuzhou 350004, China; ^2^Department of Rehabilitation at the Affiliated People's, Hospital of Fujian, University of Traditional Chinese Medicine, Fuzhou 350004, China; ^3^The Affiliated People's Hospital of Fujian, University of Traditional Chinese Medicine, Fuzhou 350004, China

## Abstract

Knee osteoarthritis (KOA) is the most common chronic bone joint disease. The WHO points out that KOA has become the fourth most disabling disease in the world, and the main clinical treatment is prevention. At present, the clinical diagnosis of knee osteoarthritis with deformation is mainly made by X-ray and two-dimensional ultrasound, and the preventive treatment effect is not good. Shear wave elastography (SWE) has been widely used in clinical practice for its advantages of noninvasive, simple, rapid, and high accuracy in soft tissue hardness. This study investigates the feasibility of using SWE in the grading diagnosis of KOA and the detection of early skeletal muscle injury. 60 patients were enrolled with unilateral KOA who met the inclusion criteria. Routine scanning and SWE exploration were carried out and compared between the affected and healthy knee joints. The measurements included morphology, damage degree of cartilage, joint effusion, joint synovial thickness, the degree of meniscus convexity, and shear wave speed (SWS) in the tendon attachment area of the quadriceps femoris superior patella, and tendon thickness and SWS between and within groups. The affected was scored according to the ultrasonic characteristics. The correlation between them was analyzed to evaluate the feasibility of SWE in grading the diagnosis of KOA. 57 cases had knee cavity effusion (57/60, 95.0%), 58 cases had knee cartilage injury (58/60, 96.6%), and 35 cases had a lateral process of the medial meniscus (35/60, 53.3%); 30 cases had synovial hyperplasia (30/60, 50%), 21 cases had osteophyte formation (21/60, 35%), and no one had a popliteal cyst. There was no significant difference in tendon thickness between and within groups (*p* > 0.05), but a significant difference in SWS (*p* < 0.01); the SWS of the quadriceps femoris tendon is negatively correlated with ultrasound score (*r* = 0.955, *p* < 0.01). There is a strong negative correlation between SWS and the degree of KOA. It can be used in the grading diagnosis of KOA to help find more early strain points.

## 1. Introduction

Unilateral knee osteoarthritis (KOA) is a common chronic degenerative disease with complex pathological changes. It is the main form of osteoarthritis disease, leading to the decline of acting ability and dysfunction of middle-aged and elderly people. The most direct symptom is pain. Its incidence is closely related to obesity, the reduction of quadriceps strength, and biomechanical pressure [1]. With the population aging and the soaring obesity rate caused by the increased prevalence of negative lifestyle choices, the disease is becoming more prevalent and is affecting younger age groups.

Shear wave elastography (SWE) is a noninvasive, quantitative, and real-time imaging of soft tissue stiffness that is considered more objective and reproducible than compression ultrasound elastography. SWE uses acoustic radiation force pulses to generate shear waves that propagate perpendicular to the acoustic beam, causing transient displacements. The shear wave velocity at each pixel is directly related to the shear elastic modulus (stiffness), which is an absolute measure of tissue elasticity. SWE is an effective method to quantify changes in muscle stiffness. Recent studies have shown that SWE can effectively measure the elasticity of neck extensors in both relaxed and contracted states.

According to the literature and previous studies, it is found that in the early stage of KOA, the hardness of soft tissue has changed without structural change [2]. Muscle stiffness is an index of muscle biomechanics. At present, gray-scale ultrasound can only make a preliminary hierarchical diagnosis of KOA from the structural aspects of synovial hyperplasia, cartilage injury, and osteophyte formation, but it cannot sensitively prompt the early injured skeletal muscle lesions. How to early detect and intervene in KOA has become a hot spot in clinical research in recent years. SWE is a new noninvasive and radiation-free technique for evaluating soft tissue elasticity. Data show that SWE shows excellent reliability and validity when evaluating muscle tissue shear modulus [3, 4].

In this study, 60 patients with early KOA with mild pain assessed by a visual analog scale (VAS) were selected, and the quadriceps femoris tendon, one of the important supporting and motor structures of the knee joint, was selected as the research point. SWE was used to evaluate the changes in shear wave speed at the attachment point of the quadriceps femoris tendon, to find the early chronic strain point of skeletal muscle, and realize the accurate early diagnosis and grading evaluation of patients with KOA.

## 2. Materials and Methods

### 2.1. Study Population

This study enrolled 60 patients with unilateral KOA in the ultrasound department, including 10 males and 50 females, with an average age of 58.3 ± 8.3 years (range 40–70 years) from May 2020 to January 2021.

Inclusion criteria were as follows: (1) consistent with the ultrasonic features of early KOA; (2) aged 40–70 years; (3) unilateral knee pain; (4) no targeted treatment; and (5) willing to sign an informed consent and participate voluntarily.

Exclusion criteria were as follows: (1) those who did not meet the ultrasonic features of early KOA or bilateral knee pain; (2) age <40 or >70 years; (3) patients with joint diseases caused by rheumatoid rheumatism, gouty arthritis, autoimmune diseases, long-term medication history, joint trauma, or operation history; (4) persons allergic to coupling agents; (5) patients with serious primary diseases such as cardiovascular, liver, kidney, digestive system, and hematopoietic system, as well as psychiatric patients; (6) there are many other medical conditions (such as kidney or liver disease or deep vein thrombosis) that hinder the participation in this study; and (7) unable to sign written informed consent.

This study and its protocols were approved by the Ethics Committee.

### 2.2. Instruments and Methods

The instrument used was the Siemens Acusonsequia512 (probe frequency 5∼14 MHz) equipped with acoustic radiation force impulse (ARFI) technology.

The patient takes the sitting position and puts a self-made pillow pad under the popliteal fossa to make the knee flexion 30 degrees [5], which stretches the extensor muscle and avoids the anisotropy caused by the depression occurring with the complete extension of the quadriceps femoris, as shown in Figure 1. Expose bilateral knee joints, apply ultrasound gel directly on the surface of the knee joints, and probe and scan slowly and carefully.

### 2.3. Scanning Steps

(1) Routine scanning of the knee joint under musculoskeletal ultrasound mode: the scanning contents include suprapatellar bursa, patellar tendon, quadriceps femoris tendon, knee cartilage, joint synovium, meniscus, ligament, etc., and the morphology, thickness, degree of wear cartilage, joint cavity effusion, joint synovium thickness, ligament morphology, etc., were recorded
  1. The quadriceps femoris tendon is the softest when the knee is flexed at 30°. At the same time, attention should be paid to the fluid in the space because a small amount of effusion often accumulates here.
  2. Sector longitudinal cutting and scanning were performed from the inside and outside of the knee joint to observe whether osteophytes were formed at the edge of the knee joint.
  3. Bend the knee joint to the maximum angle and observe the shape, thickness, and surface smoothness of articular cartilage. Early knee osteoarthritis can be considered if the following conditions are met: a. Linear hyperechoic discontinuity and roughness on the cartilage surface, increased echo in the lesion area, slight thinning or local uplift of cartilage, and increased echo of the subchondral bone line; b. The synovium of the joint was slightly thickened (2∼4 mm), with a small amount of effusion in the articular cavity with or without osteophyte.
(2) Detection of shear wave speed of quadriceps femoris tendon: using ARFI technology in Siemens Acusonsequia512, the frequency of probe is 5–12M to enter the SWE mode. The medial and lateral areas of the quadriceps femoris tendon at 1 cm above the patella are taken as study points. The SWP at each study point on both the affected and the healthy joint was measured thrice, with the average value being recorded, as shown in Figure 2.

### 2.4. Scoring Criteria for Routine Ultrasound Observation Indexes

#### 2.4.1. The Degree of Cartilage Injury [6]

(1) Normal (0 points): the cartilage surface and subchondral bone lines are smooth, continuous, clear, and sharp, and the low-echo cords are uniform; (2) Grade I (1 point): the thickness of cartilage has no obvious change, the linear hyperechoic from the surface is discontinuous and rough; (3) Grade II (2 points): the surface of degenerative cartilage is rough, the echo in the lesion area is increased, the cartilage is slightly thinner or locally uplifted, and the echo of the subchondral bone line may be enhanced in some cases; (4) Grade III (3 points): degenerative cartilage is thinner, and the echo of the subchondral bone line is enhanced and irregular; and (5) Grade IV (4 points): complete loss of degenerative cartilage layer, exposure of subchondral bone, continuous or discontinuous subchondral bone line.

#### 2.4.2. The Standard Evaluation of Synovial Thickness [7]

(1) Normal (0 points): there was no obvious synovial thickening; (2) slight thickening (2 ∼ 4 mm) (1 point); (3) moderate thickening (5∼8 mm) (2 points); and (4) severe thickening (≥9 mm) (3 points).

#### 2.4.3. Meniscus Protrusion Reference Standard [8]

(1) Mild (1 point): the protrusion is less than 1/3 of the width of the meniscus; (2) moderate (2 points): the protruding part accounts for 1/3 to 2/3 of the width of the meniscus; and (3) severe (3 points): the protruding part is greater than 2/3 of the width of the meniscus. Other scoring criteria: (a) joint cavity effusion: yes (1 point) or no (0 points); (b) osteophyte: yes (1 point) or no (0 points); and (c) popliteal cyst: yes (1 point) or no (0 points).

### 2.5. Statistical Analysis

SPSS 20.0 statistical software was used for statistical analysis. Continuous variables were statistically described by (*x* ± *s*). A two-paired sample *t*-test was used to compare the mean of the two groups, and the paired *t*-test was used to compare the mean of the same group before and after treatment. The difference was statistically significant (*p* < 0.05). The correlation between ultrasound score and shear wave speed was statistically analyzed by the Spearman correlation, *p* < 0.05, which was statistically significant. The correlation coefficient *R* was taken as an absolute value. *R* < 0.3 had no correlation, *R* > 0.3 had weak correlation, 0.3 < *R* < 0.5 had low correlation, 0.5 < *R* < 0.8 had significant correlation, and *R* > 0.8 had high correlation.

## 3. Results

### 3.1. Gray-Scale Ultrasound Features of 60 Knees with KOA

When we examined the gray-scale ultrasound features of the knees in 60 patients with KOA, we found that 57 cases affected the knee joint disability (57/60, 95.0%); 56 cases with cartilage injuries in the knee joint (56/60, 93.3%); four of them at 0 grade (4/60, 6.7%); the proportion of I degree was the largest, with 50 cases (50/60, 83.3%); while those of II degree had 6 cases (6/60, 10.0%). When we performed gray-scale ultrasound feature analysis of the lateral meniscus at the medial aspect of the knee joint in 35 (35/60, 53.3%) patients among the 60 patients with KOA, we found that 0 degrees had 25 cases (25/60, 41.7%); mild degree had 29 cases (29/60, 43.3%); moderate degree had 6 cases (6/60, 11.7%); and none were in severe stages.

When we analyzed 30 patients (30/60, 50%) with knee synostosis, it was found that 0 degrees had 30 cases (30/60, 50%); mild degrees had 30 cases; and none were in the moderate stage.

Similarly, we also found that there were 21 cases of knee osteophytes (21/60, 35%) and 0 popliteal cysts in the knee joint. Ultrasonic scoring results: 34 cases with an ultrasonic score ≤3, 26 cases with 4–6, and 0 cases with ≥7. These cases are divided into mild groups and moderate groups, respectively.

### 3.2. Comparison of Tendon Thickness and Shear Wave Speeds in Different Observation Areas

There was no significant difference in the thickness of the tendon in the medial and lateral areas of the quadriceps femoris attachment of the patient's knee joint (*p* > 0.05). The shear wave speed in the medial area was less than that in the lateral area, and the difference was statistically significant (*p* < 0.01), as shown in Table 1.

There was no significant difference in the thickness of the tendon between the medial area of the quadriceps femoris attachment on the patient's knee and the medial area of the quadriceps femoris attachment on the healthy side (*p* > 0.05). However, the shear wave value of the affected side was significantly lower than that of the healthy side (*p* < 0.01), as shown in Table 1.

### 3.3. Correlation between Shear Wave Speed of Quadriceps Femoris Tendon and Ultrasonic Score

The pain points of 60 patients with unilateral KOA occurred in the medial area attached to the quadriceps tendon, of which 5 cases were combined with the lateral area. The correlation between the shear wave value of the medial condyle and the ultrasonic evaluation score was analyzed. It was found that the shear wave value was negatively correlated with the ultrasonic score (*r* = 0.9 55, *p* < 0.01), as shown in Figure 3.

## 4. Discussion

Rheumatism is an autoimmune, allergic disease. Knee osteoarthritis is a condition in which there are abnormalities in bone metabolism, so knee osteoarthritis is not rheumatic. Its diagnostic criteria are joint pain while walking, which is especially severe when going up and down stairs; joint allodynia on physical examination; and symptom onset for more than one month. For the coccal leg, the pain is on the outside of the knee, and for type O, the pain is on the inside of the knee. From the imaging examination, it can be observed that the joint space on one side of the patient is narrower, showing osseous hyperplasia.

Guo et al. (2016) found increased tension in the trapezius muscle in patients with cervical scapular fascial pain, and SWE could detect a higher shear modulus of the trapezius muscle than normal subjects. Mitsuhiro Masaki, Tomoki Aoyama, et al. found that HCWs with low back pain had lower back muscle stiffness. SWE found that the multifidus elastic modulus in the lower back pain group was higher than that in the asymptomatic group. They suggested that back pain was associated with multifidus stiffness. In the clinic, we found that some KOA patients had knee back stiffness, traction pain, and limited mobility.

Among the many causes of KOA, the biomechanical imbalance of the knee joint is an important mechanism leading to KOA [9], which is consistent with the idea of the clinical treatment scheme. A 5-year multicenter osteoarthritis study [10] showed that quadriceps function was associated with an increased risk of worsening knee pain in women. Patients with KOA will have structural changes such as quadriceps femoris muscle fiber atrophy and increases in intramuscular fat and subcutaneous fat. The occurrence and development of KOA and its limitations on motor function are often related to the degree of key muscle injury during knee joint activity [11]. Therefore, quadriceps femoris injury is the root cause of functional limitation in patients with KOA and a major factor determining motor function. The tendon is a kind of viscoelastic tissue, which can bear the traction of external forces such as muscle contraction and produce the corresponding deformation to realize its specific biological function. The elastic value of the tendon will change to varying degrees under the conditions of degeneration or injury. Tendon lesions mainly refer to the degeneration and disintegration of collagen structures, which are related to the changes in protein and water content, cell proliferation, fat infiltration, and neovascularization [12]. In this study, the knee joint was flexed at 30° and was in the most relaxed state. The tendon deformation caused by the traction of the quadriceps femoris was excluded, and only the strain of the tendon caused by normal knee joint activities was concerned.

The 60 patients with unilateral KOA enrolled in this study all had mild pain according to VAS evaluation. The symptoms of persistent pain in the knee joint appeared in all the patients' history for almost half a year. In Gray-scale ultrasound, the echo of cartilage in the knee joint was enhanced and less smooth, and synovial hyperplasia, joint cavity effusion, meniscus convexity, or osteophyte were seen. The Gray-scale ultrasound uses the quantitative evaluation of the above contents to grade the diagnosis of KOA. Although this scoring method is objective and comprehensive, it can only score the KOA with obvious degenerative changes [13, 14].

Does KOA exist before these characteristic structural lesions? The author found that 4 cases had obvious pain symptoms, but there were no abnormal gray-scale ultrasound findings [15]. Modern life has produced many negative habits, such as prolonged exposure to cold air and inactive lifestyles, which lead to weight gain. Many overweight young people have experienced nonspecific knee pain, which has generally been considered “rheumatism” in Chinese culture. At this time, the SWE speed of the quadriceps femoris tendon has been significantly reduced, indicating that the hardness of the tendon has changed; that is, the structural components such as collagen in the tendon have changed [16, 17]. The gradual change of tendon composition will inevitably lead to the change of its function, resulting in the abnormal mechanical function of quadriceps femoris, the change of motion support effect of quadriceps femoris on the knee joint, and the change of mechanical trajectory of the knee joint, which all occurred before the obvious lesion of the knee joint structure. Pain is the earliest signal released by KOA [18–20]. Some scholars believe that the change in internal stress on the knee joint leads to synovitis, and the injured synovial cells release inflammatory mediators and matrix-degrading enzymes into the joint cavity, causing the joint to experience feedback and progressive joint degeneration. The peripheral receptors of the knee joint can cause central sensitization through pathological changes such as synovitis and subchondral bone and then lead to changes in the plasticity of central pain conduction neurons to cause neuropathic pain. The horizontal rotational motion of the tibiofemoral joint is centered on the medial condyle. Therefore, the clinical lesions of KOA are often more serious on the medial side. This was also significantly reflected in this study. All 60 patients with KOA had pain in the medial area of the knee, including 5 cases with pain in the lateral area, and the shear wave speed of the medial knee was significantly less than that in the lateral area [21, 22]. Then the correlation analysis between the shear wave value of the medial area and the ultrasonic score of the knee joint shows that the shear wave value of the affected knee joint is negatively correlated with the ultrasonic score; that is, with the increase of the score value, the shear wave speed decreases accordingly, which lays a foundation for the graded diagnosis of KOA by shear wave elastic imaging [23].

From this study, we observe that SWE is highly sensitive and the shear wave speed is decreased from an interesting point. Therefore, we propose that the point where the SWS in the sensitive area of the affected side of early KOA decreases may be the early strain point of KOA. This study also followed up the comparison of SWE values in the same parts of patients treated with acupuncture in the later stages. It was found that the pain disappeared and the SWE value increased significantly after three acupuncture treatments. Therefore, we conclude that SWE can be a good evaluation method for early strain points of KOA, guide clinically effective intervention, and prevent or delay the progress of KOA.

In this study, SWE technology was used to quantitatively evaluate the shear wave speed of the quadriceps femoris tendon in patients with KOA. However, in clinical practice, the tissue hardness information reflected by ultrasonic elastography is not always true, and its measurement results are affected by many factors. Further research can be done to compare the effectiveness of SWE in a clinical setting with the current gold standard.

## 5. Conclusion

SWE is a good method to detect soft tissue damage. There is a strong negative correlation between SWS and the degree of KOA. It can be used in the grading diagnosis of KOA to help find more early strain points.

## Figures and Tables

**Figure 1:** Check posture and a self-made pillow.

**Figure 2:** The average speed taken from the shear wave speed measured in the same study point three times, and the measurements of the three times shear wave speeds were very close.

**Figure 3:** Linear correlation between median shear-wave speed and ultrasonic scores.

**Table 1:** Comparison of tendon thickness and shear wave values within and between the groups.

Index	Affected side and healthy side				*p*
	Range	SD	Range	SD	
The thickness of the tendon inside (mm)	4.0∼6.0	5.27±0.36	4.1∼6.0	5.32 ± 0.34	0.128
	4.1∼6.1	5.32±0.34			
*p*		0.101			

SWV inside (m/s)	1.0∼5.0	3.40 ± 0.96	3.0∼8.8	6.84 ± 1.05	≤0.001
SWV outside (m/s)	1.9∼5.1	3.64 ± 0.90			
*p*		0.008			

## Data Availability

The simulation experiment data used to support the findings of this study are available from the corresponding author upon request.
